RETRACTED

# Effect of Hospital-Family Rehabilitation Intervention on Walking Function and Lower Limb Surface Electromyography in Children with Cerebral Palsy

**DOI:** 10.1155/2022/7034670

**Published:** 2022-06-08

**Authors:** Jing Wang, Ling Yue, Zhihong Chen, Bing Bai, Cuiying Chen

**Affiliations:** ^1^Department of Neurorehabilitation, Hebei Children's Hospital, China; ^2^Nursing Department, Hebei Children's Hospital, China

## Abstract

**Objective:**

To explore the effect of hospital-family rehabilitation intervention on walking function and lower limb surface electromyography in children with cerebral palsy (CP).

**Methods:**

About 100 children with CP treated in our hospital from February 2019 to April 2021 were enrolled. The patients were randomly assigned into control group and study group. The control group received routine intervention, and the study group received hospital-family rehabilitation intervention. The intervention effect, GMFM88 scale score, IMMG value, CR value, lower limb surface EMG value, and compliance of gastrocnemius muscle and tibialis anterior muscle were compared.

**Results:**

First of all, we compared the intervention effects. In the study group, 43 cases were markedly effective, 5 cases were effective, 1 case was improved, 1 case was ineffective, and the effective rate was 98.00%. In the control group, 22 cases were markedly effective, 14 cases were effective, 7 cases were improved, 7 cases were ineffective, and the effective rate of 86.00%. The intervention effect of the study group was better compared to the control group (*P* < 0.05). Secondly, we compared the scores of the GMFM88 scale. The scores of D area and E area and total score of the study group were higher compared to the control group (*P* < 0.05). The IEMG values of gastrocnemius muscle and tibialis anterior muscle were compared, and the IMMG values of passive and active gastrocnemius muscle and tibialis anterior muscle in the study group were higher compared to the control group (*P* < 0.05). There exhibited no significant difference in CR value before intervention (*P* > 0.05). After intervention, the CR values of gastrocnemius muscle and tibialis anterior muscle in the study group were significantly lower compared to the control group (*P* < 0.05). In terms of the surface EMG of lower limbs, the EMG value of passive activity (gastrocnemius muscle, tibialis anterior muscle) in the study group was higher compared to the control group, and the EMG value of active activity was significantly lower compared to the control group (*P* < 0.05). Finally, we compared the compliance. In the study group, there were 43 cases of complete compliance, 7 cases of compliance, and 0 cases of noncompliance, with a compliance rate of 100.00%. In the control group, there were 32 cases of complete compliance, 11 cases of compliance, and 7 cases of noncompliance with a compliance rate of 86.00%. The compliance rate of the study group was better compared to the control group (*P* < 0.05).

RETRACTED

**Conclusion:**

The intervention of hospital-family rehabilitation model is helpful to improve the self-care ability, cognitive function, and daily activities of children with CP, enhance the walking function and lower limb surface electromyography of children with SCP, and strengthen their qualities of life.

## 1. Introduction

Cerebral palsy (CP) is a nonprogressive brain injury syndrome caused by various reasons, which mainly occurs before or within one month after birth, including central motor limitation and postural developmental disorders [1]. At present, the incidence of infantile CP in China is about 1.8‰~4.0‰, of which spastic cerebral palsy (SCP) is the most common, accounting for 60%-70% [2]. Globally, the prevalence rate of CP varies with region, race, age, genetic variation factors, and diagnostic severity [3]. According to the data published in developed countries from 1950 to 1983, the prevalence rate of CP was 1‰~4‰; however, recently, many studies have indicated that the prevalence rate of CP is decreasing year by year [4]. The data from the Danish CP registry confirmed this conclusion. The prevalence rate of CP decreased from 2.1‰ in 1999-2001 to 1.8‰ in 2005-2007. This may be related to the launch of multidisciplinary productive science and technology training for neonatal resuscitation in Denmark in 2003 [5]. According to previous reports, the prevalence rate of CP in China is 1.8‰~6‰ [6]. The results of a survey in six provinces (autonomous regions) in China from 1997 to 1998 indicated that the prevalence rate of CP in children aged 1-6 years old was 1.92‰ [7]. However, with the rapid development of perinatal medicine, neonatal emergency medicine, and the establishment of NICU, the survival rate of some low birth weight and premature infants has been enhanced, but the prevalence of CP has also increased. In a sample survey of children with CP in Foshan, Guangdong Province, in 2015, the prevalence rate of CP between 0 and 6 years old was 2.09‰ [8]. The prevalence rate of CP in children aged 1-6 years old in five cities of Hunan Province was 2.75‰ [9]. The epidemiological survey of children with CP conducted in Hainan Province from 2015 to 2016 indicated that the prevalence rate of CP between 0 and 6 years old was 2.11‰ [10]. According to this, the prevalence rate of CP in China is higher compared to western countries, and the number of children with CP in China is also at the growth stage. Therefore, the rehabilitation of children with CP in China has a long way to go.

RETRACTED

Children with CP usually cause a series of motor dysfunction due to abnormal muscle tone, uncoordinated muscle strength, and limited joint activity, the most common of which is walking dysfunction [11]. For a long time, the clinical treatment of abnormal walking function has focused on the improvement of lower limb muscle strength and muscle tension, or correcting its abnormal posture by training. It is found in clinic that the children's motor abilities such as standing and walking have been enhanced; however, there are often some conditions such as standing instability, poor walking ability, walking instability, and easy to fall, which may be related to the poor core control ability of the children. It directly restricts its balance and coordination ability. Many clinical studies have indicated that it enhances the core stability of children with CP and effectively strengthens their walking ability [12]. However, at present, exercise training is mostly adopted to promote the core stability of children with CP, because the training requires more active cooperation of the tested children, while the children with CP lack initiative and coordination because of poor cognition and understanding. There may be a gap between the treatment effect and the expected effect. In recent years, with the development of perinatal and neonatal medicine and the wide application of neonatal intensive care unit, the incidence of elderly parturient and high-risk infants in the second-child policy has increased, and the prevalence rate of CP has an upward trend [12, 13]. There is no radical cure for CP, long-term rehabilitation treatment can reduce the degree of disability, and CP and rehabilitation costs are high; most children cannot get effective rehabilitation. The rehabilitation of CP in China is mainly hospital and community rehabilitation, and the time of community rehabilitation is short, and only a few big cities are used as pilot sites [13]. At present, the rehabilitation of children with CP is gradually transferred from the hospital and rehabilitation center to the community and family. How to ensure that the rehabilitation training is consistent with the orderly and coordinated rehabilitation training in the hospital and how to make family rehabilitation training systematic and scientific are the current research focus [14]. CP is the most common physical disability in children. The recent and widely used definition of CP is “a group of permanent motor and postural developmental disorders that lead to limited activity, attributed to nonprogressive disorders that occur in the brain of a developing fetus or infant.” Motor disorders in cerebral palsy are usually accompanied by sensory, perceptual, cognitive, communication, and behavioral disorders, epilepsy, and secondary musculoskeletal problems. Although considerable progress has been made in understanding the antecedents and prevention strategies of CP over time, little is known about our ability to determine the prognosis of CP according to the type and severity of daily function, especially when resources are scarce. Family is the main place of rehabilitation training for children with spastic cerebral palsy, and the participation of family members is of great significance to promote the rehabilitation of children, but how to increase the participation of family members and improve the professional rehabilitation training of family members is the focus of clinical research. Family rehabilitation nursing model is a family-centered rehabilitation training model, which can guide family members to fully recognize the importance of disease self-management and clarify the consequences of disobeying doctor's instructions, so as to establish a perfect family support system. Guide family members to participate in children's rehabilitation decision-making and provide personalized rehabilitation training programs. The family rehabilitation nursing model can carry out comprehensive rehabilitation training through a variety of ways, improve the professional skills of children's family members, enhance medical compliance, and ensure the implementation of rehabilitation training methods. The establishment of a family-centered support system can help children and their families establish a correct and positive healthy lifestyle and help them define their roles and tasks in the process of rehabilitation, especially to the young family members. Guide them step by step to avoid rushing for success; guide the older family members to correct their attitude, avoid overindulging the children, and let the children train in accordance with the doctor's advice. Based on this, this study focuses on the effects of hospital-family rehabilitation model intervention on walking function and lower limb surface electromyography in children with CP.

RETRACTED

## 2. Patients and Methods

### 2.1. General Information

This paper included about 100 children with cerebral palsy treated in our hospital from February 2019 to April 2021. The patients were randomly divided into the control group and study group. The control group received routine intervention, and the study group received hospital-family rehabilitation intervention. There were 30 males and 20 females in the control group, and the gross motor function classification system (GMFCS) was grade I in 0 cases, grade II in 5 cases, grade III in 11 cases, grade IV in 16 cases, and grade V in 18 cases. The types of dysfunction were spastic type (*n* = 41), involuntary exercise type (*n* = 3), ataxia type (*n* = 2), hypodystonia type (*n* = 3), and mixed type (*n* = 1). The study group ranged from 1 to 9 years old, with an average of 5.96 ± 0.58 years old. There were 32 males and 18 females. Gross motor function classification system (GMFCS) is as follows: grade I (*n* = 0), grade II (*n* = 0), grade III (*n* = 14), grade IV (*n* = 20), grade V (*n* = 16), spastic type (*n* = 36), involuntary movement type (*n* = 7), ataxia type (*n* = 1), hypodystonia type (*n* = 3), and mixed type (*n* = 3). There was no statistical significance between the two groups in general data. This study was approved by the Medical Ethics Society of our hospital, and all patients signed informed consent forms.

Diagnostic criteria are as follows: western medicine diagnostic criteria: refer to the diagnostic criteria of SCP according to the Chinese guidelines for the Rehabilitation of CP (2015); diagnostic criteria of traditional Chinese medicine: the diagnosis of CP according to the interpretation of Clinical diagnosis and treatment guidelines of traditional Chinese Medicine Pediatric Diseases (2015) [15].

Selection criteria are as follows: (1) patients with the age from 1 to 12 years old, regardless of sex; (2) no joint fixed contracture; (3) patients who can walk more than 5 meters independently without aids; (4) patients who can correctly accept action instructions; and (5) guardians agree to treatment and sign informed consent.

Exclusion criteria are as follows [16]: (1) modified Ashworth spasm rating scale score ≥ grade III; (2) patients who had received botulinum toxin or surgical treatment in the past six months; (3) patients with congenital genetic metabolic diseases or epilepsy and other nervous system diseases; (4) patients with severe basic diseases; (5) patients with visual and auditory impairment affected rehabilitation evaluation; and (6) those who could not cooperate with the completion of the scale and surface EMG test.

Elimination and shedding criteria are as follows: (1) those who interrupted treatment or choose other treatment during the trial; (2) those with incomplete test data or lack of main indicators or obviously incomplete data; (3) the occurrence of hematoma, infection, and other unexpected events need to be terminated after evaluation; and (4) deterioration of the condition or other complications.

### 2.2. Treatment Methods

Children with CP in the control group were given routine hospital intervention, and their parents were given monthly health education on CP-related knowledge. According to the results of rehabilitation evaluation, rehabilitation physicians formulate rehabilitation programs, rehabilitation therapists carry out rehabilitation training for children, parents take care of children in the usual way, and when they do not make special requirements, they take the initiative to consult or learn rehabilitation skills and give appropriate guidance. Routine rehabilitation training of integrated traditional Chinese and western medicine includes physiotherapy (PT), occupational therapy (OT), and massage.

RETRACTED

The research group accepted the intervention of hospital-family rehabilitation model: First, the hospital-community-family three-dimensional rehabilitation network was established among general hospitals, community health service centers, and families. The enrolled children with brain pain received rehabilitation treatment in three stages. One treatment cycle was 6 months. The hospital-community-family rehabilitation group completed one month of hospital rehabilitation and two months of community rehabilitation, and the parents conducted rehabilitation training in the family environment for the remaining three months.

Hospital rehabilitation stage is as follows: Children with CP were first treated in a general hospital or rehabilitation training center. At this stage, the equipment was relatively complete, and the division of labor among therapists was clear. The children completed their first evaluation here and underwent clinical rehabilitation for a period of 1 month. After the end of this stage of treatment, the rehabilitation of the children was evaluated again, and the follow-up treatment plan was determined, which was used as a reference for the follow-up community and family rehabilitation phase.

Community rehabilitation stage is as follows: The community rehabilitation staff evaluated the children, and combined with the rehabilitation program of the general hospital, the children were trained for 2 months. The children were evaluated before and after treatment, and the parents were trained in rehabilitation techniques in order to prepare for family rehabilitation in the later stage. The training for the parents of children should have a unified training standard, and the training content was the basic rehabilitation training techniques, such as the Bobath technology, Voita technology, guided education, OT, and traditional rehabilitation treatment technology. The total training time was 20 days, one hour a day, and a simple assessment was carried out on them. During this period, the patient's condition was unstable or recurrent and could be transferred to a general hospital for rehabilitation treatment.

RETRACTED

Family rehabilitation stage is as follows: the parents of the children received simple family rehabilitation training according to the training contents received in the community. During the three-month training cycle, the community staff made a unified return visit once a month and put forward suggestions on the training methods during this period. After the treatment, the children's function was evaluated by the community staff.

### 2.3. Observation Index

#### 2.3.1. Evaluation Standard of Curative Effect

There is no unified evaluation standard of the curative effect, and this subject refers to the evaluation standard of curative effect of infantile CP put forward by Ma Ruofei et al. [17]: markedly effective: the total score is increased by more than 20 points; effective: the total score is increased by 10-19 points; progress: the total score is increased by 5-9 points; and ineffective: the total score is increased by less than 5 points.

#### 2.3.2. Gross Motor Function Assessment Scale-88 (GMFM-88)

GMFM-88 is one of the most widely used scales in clinical gross motor function assessment, which is assigned into five functional areas [18]. In this subject, 39 points were enrolled for functional areas related to the lower limb walking function (13 items) and 72 points for walking areas (24 items). Every score was calculated before and after treatment, and the original total score of the two scores was calculated (111 points).

#### 2.3.3. Surface EMG Data (IEMG, CR)

Experimental instrument is as follows: Flex Comp InfinitiSA7550 surface electromyography (produced by Thought technology Company of Canada). The specific process of evaluation is as follows: (1) preparation before testing: the testing environment should be kept clean and quiet, and parents should appease their children's emotions before testing so that they can cooperate with the test later. People present try to keep quiet and mute their cell phones to reduce noise interference. Before the start of the test, use disposable alcohol cotton balls to wipe and clean locally, and if necessary, medical sponge sand can be used to remove the hair and horniness of the tested parts, in order to reduce resistance. Then input the basic information of the tested children into the system; (2) electrode placement: referring to the relevant literature, combined with the anatomical structure of tibialis anterior muscle and gastrocnemius muscle, the electrodes were placed on the tibialis anterior muscle (the ventral eminence of the lateral muscle) and the medial gastrocnemius muscle (the fullest part of the medial muscle). Two muscles of the affected limbs were enrolled from the hemiplegic children, which were two electrodes of An and B, and two electrodes of the lower extremities of the children with diplegia, which were four electrodes of A, B, C, and D, respectively; and (3) testing methods: explain the whole process of testing and related matters needing attention to the family members of the children in detail before the test, so as to facilitate the completion of the test. The resting state test is as follows: the child lies on his back on the test bed with his hands on both sides of the body. With the assistance of the child's family, keep the child in a quiet state as far as possible. Of note, the tester first observed the EMG signal displayed on the computer screen. After the signal was stable, they began to record the EMG signal of the tibialis anterior muscle and gastrocnemius muscle in the resting state of 20 seconds. Passive contraction detection is as follows: (1) passive activity detection of tibialis anterior muscle: in the supine position of the child, the detection system was adjusted to the passive stretch state. After the EMG signal was stable, the tester fixed the knee joint of the affected limb in one hand to prevent its flexion. Hold the maximum speed of the dorsum of the foot in one hand to make the metatarsal flexion to the maximum angle, and maintain it for 5 seconds, then relax for 5 seconds, and repeat the above steps 3 times; (2) passive activity detection of gastrocnemius muscle: in the supine position of the child, the detection system was adjusted to the passive stretch state. After the EMG signal was stable, the tester fixed the knee joint of the affected limb in one hand to prevent its flexion, held the fastest speed of the sole of the foot in the other to make its back flexion to the maximum angle, and maintained it for 5 seconds, then relaxed for 5 seconds, and repeated the above steps 3 times. Active contraction detection is as follows: (1) active activity detection of tibialis anterior muscle: in the supine position, the detection system was adjusted to the active stretch state. After the EMG signal was stable, tell the child to do ankle dorsiflexion to the maximum angle, maintain it for 5 seconds, then relax for 5 seconds, and repeat the above steps for 3 times; (2) active activity detection of gastrocnemius muscle: in the supine position, the detection system was adjusted to the active stretch state. After the EMG signal was stable, tell the child to do ankle plantar flexion to the maximum angle, maintain it for 5 seconds, then relax for 5 seconds, and repeat the above steps 3 times. Detection of resting state after contraction is as follows: the EMG of tibialis anterior muscle and gastrocnemius muscle in 20 seconds resting state were recorded. After the test, the system would automatically analyze the results. In the process of testing, if the child had obvious crying and resistance, which affected the test, let him rest until the mood was stable, and then test again.

RETRACTED

#### 2.3.4. Compliance

Statistics of patients include compliance, assigned into, very compliance, compliance, and noncompliance.

### 2.4. Statistical Analysis

The test results were analyzed by SPSS 22.0. The measurement data in accordance with normal distribution were expressed as *x̅*±*s*, the two independent sample *t*-test was adopted for comparison between groups, and the paired sample *t*-test was employed for self-comparison. If it did not conform to the normal distribution, it is described by the median or quartile, and the comparison between groups was described by the nonparametric test. The counting data were compared by the *χ*^2^ test. The test level was set to *P* < 0.05, which exhibited statistically significant.

## 3. Results

### 3.1. Comparison of Intervention Effect

First of all, we compared the intervention effects. In the study group, 43 cases were markedly effective, 5 cases were effective, 1 case was improved, 1 case was ineffective, and the effective rate was 98.00%. In the control group, 22 cases were markedly effective, 14 cases were effective, 7 cases were improved, 7 cases were ineffective, and the effective rate of 86.00%. The intervention effect of the study group was better compared to the control group (*P* < 0.05). All the data results are indicated in Figure 1.

### 3.2. GMFM88 Comparison of Scale Scores

Secondly, we compared the scores of the GMFM88 scale. The scores of the D area and E area and the total score of the study group were higher compared to the control group (*P* < 0.05). All the data results are indicated in Table 1.

### 3.3. Comparison of IEMG Values of Gastrocnemius Muscle and Tibialis Anterior Muscle

Next, we compared the IEMG values of gastrocnemius muscle and tibialis anterior muscle; the IMG values of gastrocnemius muscle and tibialis anterior muscle in the study group were significantly higher compared to the control group (*P* < 0.05). All the data results are indicated in Table 2.

### 3.4. CR Value Comparison

Then, we compared the CR values. Before intervention, there exhibited no significant difference (*P* > 0.05). After intervention, the CR values of gastrocnemius muscle and tibialis anterior muscle in the study group were lower compared to the control group (*P* < 0.05). All the data results are indicated in Table 3.

RETRACTED

### 3.5. Comparison of Surface Electromyography of Lower Extremities

We compared the surface EMG values of lower extremities. The EMG values of passive activities (gastrocnemius muscle and tibialis anterior muscle) in the study group were higher compared to the control group, and the EMG value of active activity (gastrocnemius muscle, tibialis anterior muscle) was significantly lower compared to the control group (*P* < 0.05). All the data results are indicated in Table 4.

### 3.6. Compliance Comparison

Finally, we compared the compliance. In the study group, there were 43 cases of complete compliance, 7 cases of compliance, and 0 cases of noncompliance, with a compliance rate of 100.00%. In the control group, there were 32 cases of complete compliance, 11 cases of compliance, and 7 cases of noncompliance, with a compliance rate of 86.00%. The compliance rate of the study group was better compared to the control group (*P* < 0.05). All the data results are indicated in Figure 2.

## 4. Discussion

CP is a group of persistent central motor and postural developmental disorders and activity limitation syndrome caused by nonprogressive brain damage in developing fetuses or infants, often accompanied by sensory, cognitive, communication, and behavioral disorders, as well as epilepsy and secondary musculoskeletal problems [19]. CP is a clinical diagnosis based on symptoms and neurological signs, and a definite diagnosis is usually made between 12 and 24 months of age, but a review of the progress in early diagnosis and treatment of CP published in JAMA Pediatrics in 2017 combs the standardized tools for early prediction of CP and clearly proposes that the time of diagnosis can be advanced to before 6 months of gestational age [20]. Study reported that the incidence of CP is 1‰~5‰ in the world, 2‰~3‰ in developed countries, and 1.8‰~4‰ in China [21]. CP is the most common physical disability in children, with 2.1 cases per 1000 cases in high-income countries [22]. In Sweden and Norway, a number of studies have indicated that the prevalence of CP in live births is about 2% [23]. In Australia and Europe, the prevalence rate is declining [24]. In low- and middle-income countries, due to the higher burden of infectious diseases and differences in prenatal and perinatal care, the exact incidence of CP appears to be higher and physical disability more severe [25]. In about 80% of cases, the cause of CP is unclear, but risk factors can often be identified from the history of pregnancy, pregnancy, delivery, and late birth, and new evidence suggests that 14% of cases have genetic components.

As one of the major diseases leading to children's disability, CP demonstrates an increasing trend, and the number of cases in rural areas is much higher compared to urban areas. According to the calculation of about 20 million newborns every year, the number of new children with CP is about 36,000 to 80,000 every year [26]. The disease affects for a long time and has a serious degree of disability, which brings great pressure to the children themselves, their families, and the society [27]. At present, there is no complete cure for CP. Long-term rehabilitation can only be used to reduce the degree of limb deformity and enhance the quality of life of children with CP. The clinical types of CP in China are as follows: spastic quadriplegia, spastic diplegia, spastic hemiplegia, involuntary movement, ataxia, and mixed type [28]. Modern rehabilitation methods for CP include drug therapy, neurosurgical treatment, orthopedic surgery, stem cell transplantation, PT, OT, wax therapy, music therapy, hydrotherapy, transcranial magnetic stimulation, hyperbaric oxygen, and sensory integration training. The rehabilitation of CP is a long-term and continuous process. The family burden of the children increases, which affects the prognosis because of economic problems and other factors that are difficult to carry out early intervention actively [29]. The community rehabilitation system in some countries is relatively perfect, and rehabilitation institutions for CP are set up in the community to provide rehabilitation and education for children. For example, the United Kingdom, as a country with relatively perfect social security, has set up special schools for children with CP, and professional therapists provide services every month [29]. A treatment center for CP has been established in the capital of Denmark, focusing on the assistance of children [30, 31]. Family rehabilitation in the United States and Britain requires a family health care model that combines hospitals and families, emphasizing the treatment of the family as a unit [32]. The rehabilitation of children with CP in China is mainly in hospitals and communities. Hospital rehabilitation equipment, facilities, professional training are mainly concentrated in big cities and high fees; although children's community rehabilitation has been developed for many years, it has not yet been popularized, especially in remote areas and rural areas. With regard to the international advanced level, there is still a big gap, and how to develop community rehabilitation is still an arduous task and challenge [33].

RETRACTED

In the rehabilitation treatment of children with CP, the rehabilitation measures are carried out separately rather than integrated in various disciplines, the children are not treated as “whole people,” and the actual participation of parents is ignored [34]. Guided education, also known as the Peto method, has become one of the most popular rehabilitation methods for children with CP because of its integrated learning concept of not being separated from the group, daily life, and emphasizing people-oriented. Its characteristic is to maximize and stimulate the learning interest of children with CP, encourage and guide them to think actively, and make use of environmental facilities and learning practice opportunities to induce learning motivation [34, 35]. Community rehabilitation is an important means to initially achieve the goal of “rehabilitation services for all” for persons with disabilities in 2015. It has the characteristics of low investment, wide coverage, and strong accessibility, but according to the survey, only 16.7% of patients with rehabilitation needs can get rehabilitation services [35]. The form of community rehabilitation in China is single, which only provides some convenient support for patients with rehabilitation needs, such as community health service centers, community rehabilitation stations, or township health centers, and shares part of the rehabilitation work of the hospital. Community rehabilitation stations are generally not equipped with professional rehabilitation teams; rehabilitation medical equipment is not as complete as general hospitals or rehabilitation centers, so the rehabilitation effect cannot achieve the best [36]. However, the cost is relatively low and close to the children, so there is no need to pay additional expenses in addition to the rehabilitation medical expenses. As far as the current situation of community rehabilitation in China is concerned, community health service centers or community rehabilitation stations can only provide parents with some guidance on professional skills and the update of the latest theoretical knowledge. However, long-term continuous rehabilitation training still depends more on family rehabilitation [37].

Family rehabilitation is the most suitable and economical rehabilitation model for children with CP in China, but the effect level of family rehabilitation for children with CP varies greatly. Because this model cannot implement systematic management like institutional rehabilitation, the relativity of dependence is poor [38]. The main influencing factors of family rehabilitation treatment dependence of children with CP are family financial burden, parents' awareness of the disease, parents' skepticism about the effect of family rehabilitation, and poor mental health of the family. Many families are unable to provide continuous treatment for children, resulting in poor dependence on family rehabilitation treatment [39]. There is a positive correlation between parents' awareness of the disease and the dependence of rehabilitation treatment. According to the survey, the higher the educational level of the parents, the higher the dependence on treatment. CP rehabilitation treatment cycle is long; if the parents of children implement family rehabilitation, the effect is too hasty and poor and cannot meet the inner expectations of children's parents, and they will be skeptical about the effect of family rehabilitation or even give up [40]. Because the parents of children with CP are in the mood of anxiety and helplessness for a long time, they are not clear about the purpose and significance of the final rehabilitation treatment, so they have a negative attitude towards the rehabilitation of children over time, which affects the dependence of family rehabilitation [41]. In family rehabilitation, parents are the main caregivers and executors of rehabilitation treatment. It is of great significance to strengthen psychological counseling to children's parents and popularize the knowledge of CP diseases for the continuation of family rehabilitation dependence, so as to promote the rehabilitation effect of children and improve the quality of life [42]. The hospital-community-family rehabilitation model refers to the establishment of a hospital-community-family three-dimensional rehabilitation model, which is an economic and effective modern rehabilitation model, which provides a top-down three-dimensional rehabilitation service for children with CP [43]. This model is based on grass-roots community health service institutions, integrates hospital rehabilitation, community rehabilitation, family rehabilitation, and vocational rehabilitation within the community and provides comprehensive and systematic rehabilitation services for children [44, 45]. Our research demonstrates that this model has definite curative effect and low cost and is more suitable for the rehabilitation of children with CP in our country.

RETRACTED

In summary, the intervention of hospital-family rehabilitation model is helpful to strengthen the self-care ability, cognitive function, and daily activities of children with CP and to enhance the walking function and lower limb surface electromyography of children with SCP.

## Figures and Tables

**Figure 1:** Comparison of intervention effects between the two groups.

**Figure 2:** Comparison of compliance between the two groups.

**Table 1:** Comparison of GMFM88 scale scores between the two groups (*x̅*±s, points).

Group	*N*	D zone	E zone	Total score
C group	50	26.39 ± 3.31	51.39 ± 4.56	78.96 ± 4.67
R group	50	30.96 ± 3.37	56.79 ± 4.42	87.92 ± 4.53
*t*		6.841	6.012	9.738
*P*		<0.01	<0.01	<0.01

**Table 2:** Comparison of IEMG values of gastrocnemius muscle and tibialis anterior muscle between the two groups (*x̅*±*s*).

Group	*N*	Passive activity		Active activity	
		Gastrocnemius muscle	Tibialis anterior muscle	Gastrocnemius muscle	Tibialis anterior muscle
C group	50	14.81 ± 2.45	9.39 ± 2.21	37.29 ± 3.31	34.19 ± 3.64
R group	50	18.85 ± 2.56	11.39 ± 3.89	46.67 ± 2.45	53.29 ± 3.31
*t*		8.061	3.160	16.106	27.451
*P*		<0.01	<0.01	<0.01	<0.01

**Table 3:** Comparison of CR values between the two groups (*x̅*±*s*).

Group	*N*	Gastrocnemius muscle CR (%)		Tibialis anterior muscle CR (%)	
		Before intervention	After intervention	Before intervention	After intervention
C group	50	58.39 ± 2.45	40.19 ± 2.45	43.78 ± 4.31	31.66 ± 2.57
R group	50	58.93 ± 2.56	31.67 ± 3.46	43.64 ± 4.42	27.59 ± 3.31
*t*		1.077	14.210	0.160	6.867
*P*		>0.05	<0.01	>0.05	<0.01

**Table 4:** Comparison of surface EMG of lower extremities between the two groups (*x̅*±*s*).

Group	*N*	Passive activity		Active activity	
		Gastrocnemius muscle	Tibialis anterior muscle	Gastrocnemius muscle	Tibialis anterior muscle
C group	50	14.58 ± 3.31	8.39 ± 2.21	47.19 ± 2.46	68.19 ± 3.31
R group	50	18.66 ± 3.44	11.46 ± 2.42	37.79 ± 3.44	52.39 ± 3.45
*t*		6.043	6.623	15.716	23.367
*P*		<0.01	<0.01	<0.01	<0.01

## Data Availability

No data were used to support this study.
